The article "Impact of HSP90α, CEA, NSE, SCC, and CYFRA21-1 on Lung Cancer Patients" was retracted in 2023. Reasons: signs of a paper mill; suspected computer-generated content; unreliable results or conclusions; concerns about the data.

# Impact of HSP90*α*, CEA, NSE, SCC, and CYFRA21-1 on Lung Cancer Patients

**DOI:** 10.1155/2021/6929971

**Published:** 2021-10-20

**Authors:** Wenwen Zhou, Yanhong Yang, Zhenzhen Wang, Yan Liu, Moslem Lari Najafi

**Affiliations:** ^1^Department of Oncology, First Hospital of Qinhuangdao, Qinhuangdao 066000, China; ^2^Graduate School, Hebei Chengde Medical College, Chengde 067000, China; ^3^Pharmaceutical Science and Cosmetic Products Research Center, Kerman University of Medical Sciences, Kerman, Iran

## Abstract

Lung cancer is a lethal disease, and early diagnosis with the aid of biomarkers such as HSP90*α* protein can certainly assist the doctors to start treatment of patient at the earliest and can save their lives. To analyse the diagnostic value of HSP90*α* expression in lung cancer patients by collecting data of patients through IoT devices to avoid delay in treatments, a study has been presented in this paper where the significance of HSP90*α* biomarker is highlighted in early diagnosis of patients suffering from lung cancer. The second objective of the research study is to examine the correlation between the appearance level of HSP90*α* biomarker and the clinicopathological features of lung cancer. It is also evaluated whether the changes in HSP90*α* index are indicative or noteworthy before and after surgery of lung cancer patients. An observatory study of 78 patients with lung cancer in Qinhuangdao Hospital is presented in this paper where the samples were collected from June 2018 to March 2020. Their data were collected through IoT devices used in the latest healthcare facilities of the hospital. The ELISA method was utilized to identify the level of plasma HSP90 and to analyse HSP90 levels between the lung cancer group and healthy group of people. The relationship between HSP90 and the clinical pathological features of 78 patients suffering from lung cancer was analysed. An electrochemical luminescence method was used to detect CEA, NSE, SCC, and CYFRA21-1 levels. ROC curve and box plots were used to determine the analytic value of HSP90 and other biomarkers used in lung cancer diagnosis. Forty-two patients with moderate to early stage lung cancer with surgical correction were selected, and paired sample *T* test was used to analyse HSP90 levels before and after surgery. The plasma HSP90 level of lung cancer patients was quite higher as compared to the group of healthy people as per the values depicted in the research study. Second, HSP90 levels are substantially higher in pathologic type, differentiation degree, stage, and the existence of the lung, liver, and bone metastases (*P* < 0.05). The level of HSP90 expression was largely impacted by a few factors such as sex, age, smoking, and tumour location (*P* > 0.05). The ROC value for HSP90 was 0.599, while the area under the curve of HSP90 combined with other four tumour markers was 0.915 in the presented case study, indicating the presence of lung cancer. Patients with lung cancer had statistically significant differences in HSP90 expression levels before and after surgery (*P* < 0.05). It is concluded that the expression level of plasma HSP90*α* in lung cancer patients increases remarkably; therefore, HSP90 can be used to monitor presence of lung cancer before and after surgery in the patients.

The article "Impact of HSP90α, CEA, NSE, SCC, and CYFRA21-1 on Lung Cancer Patients" was retracted in 2023. Reasons: signs of a paper mill; suspected computer-generated content; unreliable results or conclusions; concerns about the data.

## 1. Introduction

Historically, the diagnosis of individuals with lung cancer has created a dark chapter where people hardly survived out of this disease, and it is important to diagnose this disease at the early stage, so that the chances of survival can increase [1, 2]. It is inevitable to accurately identify the stage of the patients who are suffering from lung cancer as this eventually contributes to better prognosis and treatment options. Many techniques have been developed till date for the diagnosis of lung cancer at early stages or to describe the effective or current stage of the lung cancer with good accuracy [3, 4]. Lung cancer (LC) is the utmost communal malignant tumour that has affected the entire world badly in the current era, as per the global cancer statistics report. It has the utmost morbidity which is the greatest threat to humans globally [5]. It has the largest proportion of all cancer-related deaths, which is increasing every year and found to be the third most dangerous and lethal cancer next to breast cancer and followed by prostate cancer [6].

As there have been no distinctive symptoms and/or discomfort in early stages, most of the cancers are diagnosed in the middle or terminal stage [7]. Early diagnosis is very difficult because the indications of lung cancer are similar to other respiratory diseases or common colds. Therefore, biomarkers are used to diagnose lung cancer at the early stages to save human lives [8]. Lung cancer is classified as small-cell lung cancer and non-small-cell lung cancer based on the mass, form, diagnostic method, and prescribed treatment [9]. 85% of overall lung cancers belong to the non-small-cell lung cancer category. This is further divided into adenocarcinoma, squamous-cell carcinoma, and large-cell carcinoma [10]. Heat shock proteins (HSPs) are also termed as stress proteins and are known to be a group of proteins that are extremely articulated body cells which are easily stimulated by numerous physical factors such as fever, contagion, and tumour formations. Extensive research studies have been conducted on HSP expressions and their impact on human body that even vaccine development takes place on the basis of HSP expressions [11].

The article "Impact of HSP90α, CEA, NSE, SCC, and CYFRA21-1 on Lung Cancer Patients" was retracted in 2023. Reasons: signs of a paper mill; suspected computer-generated content; unreliable results or conclusions; concerns about the data.

HSP90*α* and HSP90*β* are the two HSP90 isoforms in the cytoplasm in the HSP90 family [12]. HSP90 family contributes to getting rid of the diseases by balancing unbalanced proteins in the cell [13]. HSP90 family expresses at a higher level as compared to the ordinary tissues to alarm the body about the growing diseases and formation of tumours/cancers in the body. Proteins that contribute to the cancer cell growth are MMP9, Hif-1 *α*, Her2/ErbB2, v-Src, Raf-1, AKT, EGFR, Met, etc. These proteins are the client proteins of the HSP90 family. These cells generate the process of signal transduction that transforms the healthy cells into tumour cells. Major targets for cancer therapy are inhibitors of HSP90 [14]. Research studies have revealed that the plasma levels of HSP90*α* are considerably high in lung cancer patients.

In [15], the authors devised a strategy using HS-27, for determining Hsp90 expression from tissue specimens for the diagnosis of breast cancer. Findings revealed that the HS-27 value was the highest in tumour tissues. Along with the Hsp90 expression, H-27 is also used as significant parameter for the diagnosis of breast cancer. The usage of HS-27 fluorescence in biopsy image was also highlighted in the paper. In past years [16], many studies have revealed that Hsp90 plays a remarkable role in determination of cancer cells and its values correlate with the presence of lung cancer. On the other hand, Hsp90 protein can slow down the cell proliferation. In addition to it, Hsp90 inhibitors can be devised in the therapies to fight against lung cancer. This paper summarizes the importance of Hsp90 expression in lung cancer study. HSP90 is a vital protein for clientele stability [17]. Therefore, HSP90 can be treated as a significant biomarker in the diagnosis and treatment of lung cancer patients. HSP90 inhibitors are developed in the recent years for producing clinical results. In this paper, the development of HSP90 inhibitors is discussed which may help in the treatment of cancer patients.

### 1.1. Major Highlights of the Paper

- This study investigates the clinical usefulness of HSP90 expressions as a biomarker of lung cancer diagnosis. It examines the correlation between the expression of the HSP90 and other clinical factors of non-small-cell lung cancer.
- This paper examines the diagnostic value of HSP90*α* for lung cancer patients by detection of HSP90*α* expression levels in the diseased patients, and comparison of HSP90 with the traditional tumour markers is also evaluated.
- The proposed study detects the expression level of HSP90*α* in peripheral blood of lung cancer patients and analyses its correlation with clinical pathological characteristics of lung cancer.
- The observational perspective study detects changes of HSP90*α* in patients before and after surgery.
- This paper uses the IoT technology for easy diagnosis of the lung cancer patients and reporting the stage of tumours for providing remedial solutions.

The article "Impact of HSP90α, CEA, NSE, SCC, and CYFRA21-1 on Lung Cancer Patients" was retracted in 2023. Reasons: signs of a paper mill; suspected computer-generated content; unreliable results or conclusions; concerns about the data.

### 1.2. Organization of the Paper

This paper is organized as follows. The paper begins with introduction about lung cancer, followed by the need to devise new mechanisms for detection of lung cancer, and then highlights the contributions of the paper and existing works in the related field. The next section discusses methods and materials. Third section presents the experimental study and outcomes. Final section concludes the proposed research work.

## 2. Proposed Methods

### 2.1. The Patients First Diagnosed with Lung Cancer in the Outpatient and Inpatient Service of Qinhuangdao Hospital

From June 2018 to March 2020, 40 plus healthy physical examinees were selected as research conductors. The 78 patients in the lung cancer group were diagnosed by pathological examination, with 53 males and 25 females, aged 31～80 years old, with an average of 61.6 ± 8.8 years, including 45 cancer cases of lung adenocarcinoma, 22 cancer cases of squamous-cell lung carcinoma, 10 cancer cases of small-cell lung cancer, and 1 case of large-cell lung cancer. Staging was performed according to the 8th edition of international TNM (tumour, node, and metastasis) staging system for lung cancer. There were 26 cases in stage I, 8 cases in stage II, 18 cases in stage III, and 26 cases in stage IV. 42 individuals with surgical reasons in the early and intermediate stages of lung cancer need to be examined for HSP90 levels before and one month after surgery. The healthy group consisted of 40 healthy physical examinees in our hospital's physical examination centre during the same period, including 24 males and 16 females, aged 24～77 years, with an average of 56.5 ± 14.4 years. Before the experiment, the patients' consent and approval by the Medical Ethics Committee of Qinhuangdao Hospital were obtained.

### 2.2. Inclusion Criteria for the Patients

The enrolled patients are pathologically diagnosed with lung cancer.

- The patients who had not received radiotherapy, chemotherapy, or targeted therapy in the first diagnosis.
- The patients who had no acute and chronic infectious diseases or autoimmune diseases.
- The patients who had no serious heart, liver, kidney, and other organ diseases.
- The patients who had no other primary malignant tumour.

The article "Impact of HSP90α, CEA, NSE, SCC, and CYFRA21-1 on Lung Cancer Patients" was retracted in 2023. Reasons: signs of a paper mill; suspected computer-generated content; unreliable results or conclusions; concerns about the data.

### 2.3. Exclusion Criteria for the Patients

- Those who were unwilling to cooperate and with mental illness.
- Those who had serious heart, brain, liver, kidney, or other organ diseases.
- Those who had other malignant tumours.
- Those who had other lung diseases.
- Pregnant women.

### 2.4. Sampling

The specimens were collected from all the patients in the morning with an empty stomach. Specimens were re-collected from lung cancer patients one month after the surgery. 5 ml of peripheral plasma was retained using EDTA-K2 anticoagulant tube, shaken well, placed in a centrifuge for centrifugation for 10 minutes with revolving speed of 3000 r/min, and stored in the refrigerator at −80°C for testing. HSP90 was detected by enzyme-linked immunoassay analyser and HSP90*α* detection kit.

### 2.5. Reference Range

The normal reference range of plasma HSP90*α* was set to 0–82.06 ng/mL, the normal value of serum CEA was set to 0–4.7 ng/mL, the normal value of NSE was 0–17 ng/mL, normal value of SCC (squamous-cell carcinoma-associated antigen) was 0–1.5 ug/L, and normal value of CYFRA21-1 (cytokeratin 19 fragment) was 0.1–3.3 ng/mL.

### 2.6. Statistical Analysis

The statistical evaluation was performed using SPSS22.0 to analyse the outcomes of biomarkers in prediction of cancer stages. The sampling data were expressed by *x* ± *s*, and *T*-test was used for showing the differences between groups of normal and diseased patients. One-way analysis of variance was performed for assessment among multiple groups with respect to biomarkers. The non-parametric test was conducted if normal distribution was not followed. The ROC curve was used to analyse the prognosis value of plasma HSP90*α* and other tumour biomarkers in lung cancer.

## 3. Results and Analysis

### 3.1. Detection Results of HSP90*α* in Serum of the Two Groups

The expression level of HSP90*α* was (92.949 ± 57.741) ng/ml in the lung cancer group and (45.876 ± 12.062) ng/ml in the healthy control group, which showed statistically significant difference (*t* = 5.089, *P* < 0.01). The more values in expression level of HSP90 indicate that the person is suffering from cancer or having tumour inside the body. The baseline HSP90 levels of lung cancer patients were expressively higher than those of the healthy group of people.

### 3.2. Analysis of the Relationships

The relationships were analysed between plasma HSP90*α* levels and clinical characteristics such as different gender, age, smoking, pathological type, degree of differentiation, staging, presence of lymph node metastasis, lung metastasis, liver metastasis, and bone metastasis in 78 lung cancer patients. The results suggested that HSP90*α* level is significantly different in terms of pathological types, degree of differentiation, staging, presence of lung metastasis, liver metastasis, and bone metastasis, showing statistically noteworthy difference (*P* < 0.05); there is no noteworthy difference in HSP90*α* expression regardless of different genders, ages, smoking, and tumour sites (*P* > 0.05), as shown in Table 1.

The article "Impact of HSP90α, CEA, NSE, SCC, and CYFRA21-1 on Lung Cancer Patients" was retracted in 2023. Reasons: signs of a paper mill; suspected computer-generated content; unreliable results or conclusions; concerns about the data.

HSP90 is an indicative parameter for the diagnosis of lung cancer, but other variables, such as gender, age, lymph node, blood report, stage, and LDH levels, were not found to be correlated with the expression level of HSP90 concentrations.

### 3.3. ROC Curve Analysis

Figure 1 depicts the ROC curve based on data from the lung cancer group and the control group for HSP90, CEA, CYFRA21-1, and SCC with lung cancer as the state variable 1. The AUC value of HSP90*α* was 0.599, while the area under the curve (AUC) value of HSP90*α* combined with the other four tumour biomarkers reached 0.915, as shown in Figure 2 and Table 2, respectively. Figure 2 reveals that all the biomarkers such as CEA, CYFRA21-1, and SCC play an important role in diagnosis of lung cancer apart from HSP90*α*, and the box plots show that the actual values of biomarkers in lung cancer patients reside within the lower and higher limits of expression levels defined for lung cancer diagnosis.

### 3.4. Comparative Analysis

The preoperative and postoperative HSP90 expression levels of 42 lung cancer patients were compared before and after surgery. The preoperative HSP90*α* expression level was 64.44 ± 28.94 ng/ml, and the postoperative HSP90*α* expression level was 37.47 ± 19.66 ng/ml, showing statistically significant difference (*t* = 4.826, *P* < 0.01). This shows that the postoperative value of HSP90*α* reduces at a noteworthy level. The lung cancer patient can feel more relieved and better after surgery as the HSP90*α* expression level of lung cancer patients comes close to the expression level of healthy group of people. However, even after surgery, the HSP90*α* level of lung cancer patients remains higher than that of the healthy group of people, but still the expression level values before and after surgery show remarkable differences.

## 4. Discussion

HSP90*α* is not secreted or secreted very low under normal physiological conditions, and when there is some abnormality in the body, then high secretion of HSP90*α* is found in the body; the abnormal conditions can be caused by stress, high fever, inflammation, hunger, tumours, or cancers in the body. It can be highly expressed in various tumour cells, such as lung cancer, liver cancer, and pancreatic cancer. HSP90*α* expression in cancer cells can be 3～11 times that of normal cells. HSP90*α* may be involved in tumour cell angiogenesis, cancer cell proliferation, infiltration, metastasis, and death. A large number of studies have shown that HSP90 overexpression is a poor prognostic factor in different types of malignant tumours [18, 19]. But recent studies and our method have confirmed that HSP90*α* could be used as a potential lung cancer diagnostic indicator, which is highly expressed in the case of late lung cancer clinical stage, large tumour volume, and lymphatic metastasis. It is found that HSP90*α* has significantly different expressions between diseased and healthy people, with higher expression in lung cancer patients with lymph node metastasis group.

The article "Impact of HSP90α, CEA, NSE, SCC, and CYFRA21-1 on Lung Cancer Patients" was retracted in 2023. Reasons: signs of a paper mill; suspected computer-generated content; unreliable results or conclusions; concerns about the data.

We have examined the association between HSP90*α* and clinical pathological parameters in surgical specimens of lung cancer patients; it is found out that HSP90*α* is clearly related to large tumour volume, obvious tumour infiltration, lymphatic metastasis, and early as well as late clinical stage of lung cancer patients. It has been discovered that HSP90*α* expression in lung cancer is significantly greater than in benign diseased patients and the healthy group (47.63 ± 14.98 ng/mL). The AUC value of HSP90*α* against lung cancer is 0.857, sensitivity is 93.10%, and specificity is 62.5%, so HSP90*α* is anticipated to become a tumour biomarker for lung cancer diagnosis. It is found that HSP90*α* is expressively higher in lung cancer patients than in healthy people (*P* < 0.001). It is also found that HSP90*α* is highly articulated in the blood of diseased patients with lung cancer where plasma content is positively correlated with malignant degree of lung cancer and can be claimed as a tumour biomarker for early screening of lung cancer.

By drawing the ROC curve of the non-small-cell lung cancer group and box plots values with lower and upper value limits of HSP90*α* and other tumour biomarkers such as CEA, CYFRA21-1, and SCC, it is found that the patients with higher HSP90*α* are at later stages. The experimental analysis shows that HSP90*α* has increased expression level in lung cancer patients, and the ROC curve suggests that apart from HSP90*α* expression levels, other four tumour biomarkers such as CEA, NSE, SCC, and CYFRA21-1 can also be tested for the optimal diagnostic efficacy. Further analysis is made on the relationship between HSP90*α* and the clinicopathological characteristics of 78 lung cancer patients: in case of last tumour stages, HSP90*α* detection level in the patient's plasma is quite high. Our research results are basically consistent with some previous literature reports [20–22]. In addition to it, in this study, HSP90*α* is tested for the first time before and after the surgery of lung cancer patients, indicating that the postoperative level is significantly lower with statistically significant difference in lung cancer patients. In summary, HSP90*α* can be used as a new tumour biomarker for analysis of the lung cancer patients; therefore, HSP90*α* can be considered as a potential biomarker for further clinical development and application in the prognosis of lung cancer patients.

The article "Impact of HSP90α, CEA, NSE, SCC, and CYFRA21-1 on Lung Cancer Patients" was retracted in 2023. Reasons: signs of a paper mill; suspected computer-generated content; unreliable results or conclusions; concerns about the data.

## 5. Conclusion

The research study in this paper is based on the detection of lung cancer and is to inform the patients whether they are next to early stage of the cancer on the basis of HSP90*α* expression. Monitoring HSP90*α* expression in lung cancer has a diagnostic utility, and data from patients are collected via IoT devices. The correlation between the expression level of HSP90*α* and the clinicopathological features of lung cancer is investigated. It is found that HSP90*α* has significantly different expressions between lung cancer and healthy people, with higher expression in lung cancer with lymph node metastasis group. It has been discovered that HSP90 expression in lung cancer is significantly greater than in benign diseased patients and the healthy group (47.63 ± 14.98 ng/mL). The area under the diagnosis curve of HSP90*α* against lung cancer is 0.857, sensitivity is 93.10%, and specificity is 62.5%, and thus HSP90*α* is anticipated to become a tumour biomarker for lung cancer diagnosis. It is found that HSP90*α* is expressively higher in lung cancer patients than in normal and healthy people (*P* < 0.001). In a nutshell, HSP90*α* can be considered as a potential biomarker for further clinical development and application in the diagnosis of lung cancer patients. In future, we will study more biomarkers that can indicate specific types of cancers and we will attempt to determine the relationship between the expression levels of the parameters and the stage of the cancer. If the research study can prove the significance of the expression levels of the biomarkers that assist in diagnosis of cancers and their respective stages, then the patients can be treated accordingly as per their respective stages of the cancers.

## Figures and Tables

**Figure 1:** ROC curves of HSP90*α*, CEA, CYFRA21-1, and SCC in the diagnosis of lung cancer.

**Figure 2:** Diagnostic efficacy of HSP90*α*, NSE, SCC, CYFRA21-1, and CEA.

**Table 1:** Correlation between plasma HSP90*α* concentration and various clinical pathological parameters of lung cancer.

Pathological feature	Number of cases	HSP90*α* (ng/ml)	*P*
Male	53	89.77 ± 55.03	0.2
Female	25	99.69 ± 63.76	0.2
Age ≥ 65	39	84.57 ± 58.52	0.4
Age ＜ 65	39	101.32 ± 56.46	0.4
Smoking—yes	41	86.61 ± 51.75	0.88
Smoking—no	37	84.77 ± 54.31	0.88
Left side	34	93.95 ± 67.03	0.8
Right side	44	92.17 ± 50.21	0.89
Adenocarcinoma	45	85.03 ± 47.87	0.5
Small cell	10	147.67 ± 47.00	0.4
Squamous carcinoma	22	78.27 ± 53.64	0.6
Giant cell	1	225.39	0.621
*Degree of differentiation (DoD)*			
High DoD	17	67.90 ± 37.57	0.608
Moderate DoD	22	81.28 ± 47.49	0.624
Poor DoD	28	90.06 ± 55.37	0.689
Undifferentiated	11	154.74 ± 67.74	0.749
1.	26	64.98 ± 38.67	0.7
2.	8	64.91 ± 15.87	0.68
3.	18	89.15 ± 47.92	0.6
4.	26	132.18 ± 66.82	0.6
Lung metastasis—yes	11	113.75 ± 69.92	0.04
Lung metastasis—no	62	80.65 ± 49.34	0.04
Lymph node metastasis (LNM)—yes	44	89.52 ± 48.38	0.081
LNM—no	35	81.26 ± 57.67	0.081
Bone metastasis (BM)—yes	14	111.38 ± 51.02	0.01
BM—no	65	81.37 ± 52.07	0.01

The article "Impact of HSP90α, CEA, NSE, SCC, and CYFRA21-1 on Lung Cancer Patients" was retracted in 2023. Reasons: signs of a paper mill; suspected computer-generated content; unreliable results or conclusions; concerns about the data.

**Table 2:** Diagnostic efficacy of HSP90*α*, NSE, SCC, CYFRA21-1, and CEA.

Tumour marker	AUC	Std	*P* value	95% confidence interval	
				Lower limit	Upper limit
HSP90*α*	0.599	0.064	0.105	0.473	0.724
NSE	0.497	0.057	0.965	0.386	0.609
SCC	0.472	0.065	0.650	0.344	0.601
CYFRA21-1	0.840	0.039	0.001	0.763	0.917
CEA	0.724	0.057	0.001	0.613	0.836
Hsp90*αα* + the above 4 markers	0.915	0.029	0.001	0.858	0.972

## Data Availability

The data used to support the findings of this study are available from the corresponding author upon request.
